The article "Application of Artificial Intelligence in Radiotherapy of Nasopharyngeal Carcinoma with Magnetic Resonance Imaging" was retracted in 2023. Reasons: signs of a paper mill; compromised peer review; unreliable results or conclusions.

# Application of Artificial Intelligence in Radiotherapy of Nasopharyngeal Carcinoma with Magnetic Resonance Imaging

**DOI:** 10.1155/2022/4132989

**Published:** 2022-02-02

**Authors:** Wanlu Zhao, Desheng Zhang, Xinjian Mao

**Affiliations:** ^1^Radiotherapy Department, Huzhou Central Hospital and Affiliated Central Hospital Huzhou University, Huzhou 313003, China; ^2^Radiology Department, Huzhou Central Hospital and Affiliated Central Hospital Huzhou University, Huzhou 313003, China

## Abstract

The value of automatic organ-at-risk outlining software for radiotherapy is based on artificial intelligence technology in clinical applications. The accuracy of automatic segmentation of organs at risk (OARs) in radiotherapy for nasopharyngeal carcinoma was investigated. In the automatic segmentation model which is proposed in this paper, after CT scans and manual segmentation by physicians, CT images of 147 nasopharyngeal cancer patients and their corresponding outlined OARs structures were selected and grouped into a training set (115 cases), a validation set (12 cases), and a test set (20 cases) by complete randomization. Adaptive histogram equalization is used to preprocess the CT images. End-to-end training is utilized to improve modeling efficiency and an improved network based on 3D Unet (AUnet) is implemented to introduce organ size as prior knowledge into the convolutional kernel size design to enable the network to adaptively extract features from organs of different sizes, thus improving the performance of the model. The DSC (Dice Similarity Coefficient) coefficients and Hausdorff (HD) distances of automatic and manual segmentation are compared to verify the effectiveness of the AUnet network. The mean DSC and HD of the test set were 0.86 ± 0.02 and 4.0 ± 2.0 mm, respectively. Except for optic nerve and optic cross, there was no statistical difference between AUnet and manual segmentation results (*P* > 0.05). With the introduction of the adaptive mechanism, AUnet can achieve automatic segmentation of the endangered organs of nasopharyngeal carcinoma based on CT images more accurately, which can substantially improve the efficiency and consistency of segmentation of doctors in clinical applications.

## 1. Introduction

Nasopharyngeal cancer is a malignant tumor, and the clinical manifestations of patients are mainly nasal congestion, blood in the nose, and hearing loss, which seriously endanger patients' life and health. At present, the common clinical treatment for nasopharyngeal carcinoma is radiation therapy, which has certain moderate sensitivity [1]. Along with radiation therapy, it is also important to give patients the corresponding rehabilitation exercise [2]. However, patients often neglect the rehabilitation exercises, and, therefore, the prognosis of patients is not satisfactory. Therefore, in this study, radiation therapy combined with temporomandibular joint exercise intervention was used for patients with nasopharyngeal carcinoma, with the aim of investigating the effect of radiation therapy and magnetic resonance imaging (MRI) signs.

The article "Application of Artificial Intelligence in Radiotherapy of Nasopharyngeal Carcinoma with Magnetic Resonance Imaging" was retracted in 2023. Reasons: signs of a paper mill; compromised peer review; unreliable results or conclusions.

Surgery, chemotherapy and radiotherapy are the three main treatment modalities for malignant tumors. Radiotherapy is the only treatment mode that can be electronic and intelligent, and it is very important to promote the development of intelligent technology of radiotherapy to improve the efficacy of tumor patients. It is very important to promote the development of intelligent radiotherapy technology to improve the efficacy of tumor patients. In recent years, with the development of computer technology and intensity modulation technology, intensity modulated radiotherapy (IM-RT) uses pen-shaped beams of different intensities to irradiate the tumor target area and adjacent important tissues at different doses and precisely outlines the tumor target area and organs at risk (OARs). The precise contouring of tumor target areas and organs at risk (OARs) is a prerequisite and guarantee for precise radiation therapy. Radiotherapists need to precisely map the target areas and OARs on CT images, which is often a time-consuming and laborious process involving a lot of simple and repetitive tasks. These tasks reduce the efficiency of clinical treatment [2, 3], delay patient treatment time, and impose a burden on busy clinical work. In recent years, with the development of artificial intelligence technology in the field of radiotherapy medicine, automatic outlining software such as MIM, On *Q*, and ABAS have been widely reported [4–6]. However, the accuracy of automatic outlining technology is yet to be proven, so it is necessary to conduct a more detailed and accurate study of automatic outlining technology before applying it to clinical practice.

Nasopharyngeal carcinoma is a common malignant tumor, and radiotherapy is one of its main treatment methods [1]. Intensity-modulated radiotherapy (IMRT) [2, 3] and volumetric rotational intensity-modulated radiotherapy (VMAT) [4] have gradually become common techniques for the treatment of nasopharyngeal carcinoma in the last two decades. These techniques allow to increase the dose to the target area while reducing the risk of exposure to organ-at-risk (OARs). The aim of radiation therapy planning is to ensure that the tumor receives adequate doses of radiation without exposing the organs at risk to excessive radiation damage. OARs are very sensitive to radiation, and excessive radiation exposure may cause irreversible damage to the organ. Therefore, the identification of the boundaries of the organs at risk is critical.

The article "Application of Artificial Intelligence in Radiotherapy of Nasopharyngeal Carcinoma with Magnetic Resonance Imaging" was retracted in 2023. Reasons: signs of a paper mill; compromised peer review; unreliable results or conclusions.

Currently, there is still a lack of systematic and effective guidance for the outlining of nasopharyngeal carcinoma OARs. In this paper, we used automatic image outlining software based on artificial intelligence technology to study the accuracy of outlining of nasopharyngeal carcinoma, a head and neck tumor with more endangered organs, and developed a cascading adaptive cluster network (AUnet) based on Unet. Used for automatic segmentation of organ-threatening nasopharyngeal carcinoma radiation therapy, the method not only provides fast and accurate segmentation of OARs, but also improves the segmentation of small organs in the head and neck. It adds an adaptive mechanism, which can capture organs of different sizes at different encoding and decoding layers, and calculates the convolution of the AUnet network according to the size of the organs, thus adopting a special cascade network structure to adapt to the segmentation of different organs and using its a priori information to improve the segmentation accuracy thus better meeting clinical needs.

The accuracy of automatic segmentation of organs at risk (OARs) in radiotherapy for nasopharyngeal carcinoma was investigated. In the automatic segmentation model which is proposed in this paper, after CT scans and manual segmentation by physicians, CT images of 147 nasopharyngeal cancer patients and their corresponding outlined OARs structures were selected and grouped into a training set (115 cases), a validation set (12 cases), and a test set (20 cases) by complete randomization. Adaptive histogram equalization is used to preprocess the CT images. End-to-end training is utilized to improve modeling efficiency and an improved network based on 3D Unet (AUnet) is implemented to introduce organ size as prior knowledge into the convolutional kernel size design to enable the network to adaptively extract features from organs of different sizes, thus improving the performance of the model.

The remaining paper is organized according to the following structure. In Section 2, a thorough analysis of the state-of-the-art existing methods is presented followed by materials and methodology (Section 3) used in the proposed setup described in detail. In Section 4, experimental results and observations were presented along with the effective performance of the proposed scheme in resolving the issue. A generalized discussion on both existing state-of-the-art and proposed techniques is provided in Section 5. Finally, concluding remarks are given.

The article "Application of Artificial Intelligence in Radiotherapy of Nasopharyngeal Carcinoma with Magnetic Resonance Imaging" was retracted in 2023. Reasons: signs of a paper mill; compromised peer review; unreliable results or conclusions.

## 2. Related Work

Outlining target areas and endangering organs [5], which is essentially an image segmentation task, is usually done manually by experienced physicians layer by layer. However, the manual segmentation (MS) process is time consuming [6] and the accuracy of segmentation depends on the experience of the physician. Many studies have found large differences in the segmentation results of these regions of interest (ROIs) among different physicians. Automatic segmentation of CT images [7] can significantly reduce the physician's workload and improve the accuracy and consistency of ROIs segmentation. Clinically, “template-based segmentation” (ABS) [8, 9] and “automatic template-based segmentation” (ABAS) [10, 11] are based on previous “alignment” experience. Lu et al. [13] evaluated the clinical application of ABS and showed that ABS has a high accuracy, but further analysis revealed that there are two main challenges in using ABS: first, it is difficult to build a universal template based on fixed images because the anatomical morphology of human organs often changes, and even the same ROI may vary greatly due to differences in patient size and age. The atlas-based construction of patient template images often does not take into account such differences, which makes it difficult to obtain a more accurate segmentation structure for patients with large body size deviations. Secondly, the alignment time of ABS is affected by various factors such as alignment site and range, image modality, and quality. It is often the case that clinically satisfactory alignment accuracy or results are not achieved even after spending a lot of alignment time.

In recent years, deep learning methods have been widely used. For example, stacked autoencoders (SAEs) [14], deep belief networks (DBNs) [15], restricted Boltzmann machines (RBMs) [16], recurrent neural networks (RNNs) [17], and convolutional neural networks (CNNs) [18] have become the most popular deep learning algorithms. Melendez et al. applied various learning techniques to detect chest X-ray tuberculosis with an area under the curve (AUC) of 0.86. Hu et al. proposed a liver segmentation framework based on CNN and full-surface optimization with an average similarity coefficient (DSC of 97%. Esteva et al. fed a large dataset into CNN to classify skin cancer with higher accuracy than dermatologists. CNN learned a large number of input and output mapping relationships between them to automatically extract multilevel visual features. When the convolutional network is trained by certain methods (generally by backpropagation to train the parameters of the neural network), the weights of each layer can be adjusted. Unet is an end-to-end architecture consisting of two important sampling components, which adds upsampling and downsampling processes compared to CNN. Unlike typical CNNs, Unet uses downsampling to generate images of different resolutions and convolves images of various resolutions. Information is extracted from multiple levels and synthesized when upsampling reconstructs low resolution feature images. Recently a new segmentation structure based on nested dense jump connections (Unet++) has emerged with good results for image segmentation tasks. Both Unet and DDNN use end-to-end models unlike networks with non-end-to-end models such as mask-RCNN, where the non-end-to-end model N slightly reduces accuracy, improves efficiency, and also reduces network complexity. The encoding part extracts the image features and the decoding part restores the original resolution. Unlike Unet, DDNN uses deconvolution rather than upsampling to recover the original resolution. In a recent study, Men et al. used CNN and DDNN for head and neck organ endangerment segmentation and also achieved good results.

The article "Application of Artificial Intelligence in Radiotherapy of Nasopharyngeal Carcinoma with Magnetic Resonance Imaging" was retracted in 2023. Reasons: signs of a paper mill; compromised peer review; unreliable results or conclusions.

## 3. Proposed Methodology (Materials and Methods)

### 3.1. Data Acquisition

Using a large-aperture CT simulator (Philips Medical Systems, Cleveland, Ohio, USA), CT scans were performed on patients with nasopharyngeal carcinoma according to clinical requirements with the following parameters: layer thickness 3 mm, voltage 120 kVp/140 kVp, current 300 mAs, layer spacing 3 mm, increment 3 mm, collimation 16 × 0.75 (mm), display FOV 600 mm, scan FOV 600 mm, reconstruction filter type UB/B, and pitch 0.567. OARs of patients with nasopharyngeal carcinoma were outlined by physicians at TPS and reviewed and confirmed by another senior oncologist, CT and RT structural data from our oncology control center (Sun Yat-sen University Cancer Center, SYSUCC).

A total of 147 patients were included in this paper, and after CT scans and manual segmentation by physicians, they were directly randomized and 20 patients were selected as the test set by a complete randomization method (random number method). The remaining data were randomly divided into a training set (90%) and a validation set (10%) for 10-fold cross-validation. The training set was input to AUnet for model training; then the performance of the model was evaluated using the validation set; and finally the test set was used for testing. The overall flow chart of this paper is shown in Figure 1.

### 3.2. Image Preprocessing

The final output of a deep learning-based segmentation task is closely related to the quality of the input images. Given that there are numerous OARs in CT images of nasopharyngeal cancer patients and some have similar gray values, shapes, or textures, this paper uses an image enhancement method to preprocess the input image data to improve the image contrast.

The article "Application of Artificial Intelligence in Radiotherapy of Nasopharyngeal Carcinoma with Magnetic Resonance Imaging" was retracted in 2023. Reasons: signs of a paper mill; compromised peer review; unreliable results or conclusions.

Histogram equalization (HE) is a basic method for image enhancement, and adaptive histogram equalization (AHE) is improved by histogram equalization (HE). HE improves local contrast; enhances edge sharpness in each region of the image; improves the quality of the original CT image; and improves the shape, texture, and boundary information of the organ. Before input to the network, the normalized image grayscale values are [0∼1] and the image size is 512 × 512.

## 4. AUnet Model in This Paper

In this paper, based on the Unet model, an adaptive mechanism is introduced to generate an improved network structure of AUnet for the purpose of automatic segmentation of OARs in nasopharyngeal cancer radiation therapy. The AUnet network has multiple encoder and decoder components; the encoder network is used to extract the visual features of medical images and the decoder network recovers the original resolution by deconvolution. Convolution levels at different scales focus on processing organs of different sizes. Before convolution, the image data of that scale layer is stitched with the image data of the next scale layer after upsampling. Features collected on different resolution images not only flow within the same layer, but also pass between layers (the previous layer); this design together with jump connections improves the information utilization of the network (Figure 2).

In AUnet's segmentation model, an adaptive mechanism is introduced, which is the process of automatically adjusting the processing method, processing order, processing parameters, boundary conditions, or constraints according to the data characteristics of the processed data during processing and analysis, so that they are compatible with the statistical distribution characteristics and structural characteristics of the processed data to achieve the best processing results. In the AUnet model, the encoder can capture a variety of low-level features from multiple scales, including intensity, texture, and contour raw information. At the end of decoding, global and local perceptual information of the perceptual domain is extracted from the feature images. Each encoding module learns multiple scale features by using different size filters whose sizes are calculated by the volume of the organ. Combining these multiscale features, AUnet can maintain reliable information on boundaries, textures, and shapes, greatly improving segmentation accuracy.

The size of each convolution kernel is calculated according to the volume of the organ. The edge length is obtained by (1), where *v*_*j*_ is the volume of the j-th organ, *v*_*sum*_ is the volume of the whole image, and size represents the size of the feature map of each level. A series of *r*_*i*_ can be calculated for each image, and the formula is as follows:

(1) $$\begin{array}{c} r_{i}=size_{f}.\left[\frac{v_{j}}{v_{sum}}\right]. \end{array}$$

The size of convolution kernel is related to the size of organs. In the network structure shown in Figure 2, *x*_0,0_ is the input and *x*_4,0_ is the output. In the upper part of the square network, the size of the convolution is set to be smaller in order to capture smaller organ features. In the lower part of the square network, the downsampled image has large resolution and is suitable for capturing larger organ features. Therefore, we set the size of the convolution kernel to be larger than the upper half of the relative network. The convolution kernel size is calculated according to the volume of the organ. If the number of organs is greater than the number of downsampling scale layers (*r*_*i*_ cannot be assigned to the corresponding scale layer), the smaller *r*_*i*_ is discarded.

The article "Application of Artificial Intelligence in Radiotherapy of Nasopharyngeal Carcinoma with Magnetic Resonance Imaging" was retracted in 2023. Reasons: signs of a paper mill; compromised peer review; unreliable results or conclusions.

After the network outputs the prediction image, the “open operation” is used to smooth the contour and eliminate small outliers. As shown in Figure 3, after setting the convolution kernel size of each layer, the input image has organ feature information from *x*_0,0_ to *x*_0,4_ after multiple feature extraction. *x*_0,4_ After upsampling, these feature data are accumulated with the output data of each layer, and then the feature extraction is performed again. The jump connection in Figure 3 is shown in detail in Figure 4, where *g* (*x*) represents the convolution operation, and *f* (*x*) represents the superposition operation of the convoluted result *g* (*x*) and the input data *X*.

The AUnet proposed in this study inputs CT images into the network. Before input, CT images are preprocessed to improve the definition of contour. In order to improve the efficiency of model training and realize the end-to-end training process, the trained AUnet network can segment the selected 15 organs at the same time and train an AUnet to get the results of 15 organs at the same time. We use deep learning to realize model training, evaluation, error analysis, and visualization. In the experiment, data enhancement techniques are used, such as random shear, flip, gray-scale disturbance, and shape disturbance. After that, random momentum gradient descent is used to optimize the loss function. The initial learning rate is set to 0.0001, the learning rate attenuation factor is set to 0.0005, and the attenuation step is set to 2000. When the loss function of the verification set is no longer reduced, we no longer use the fixed step training model until the average accuracy of the training set ends for segmentation. UNET, AUnet, and DDNN all adopt end-to-end models. Different from non-end-to-end models such as mask RCNN, their accuracy is slightly reduced, efficiency is improved, and network complexity is reduced. In each coding and decoding layer, adaptive convolution kernel operation is added to calculate the size of convolution kernel according to the volume of organs in each layer. The network can extract organ features of different sizes from images with different resolutions.

The article "Application of Artificial Intelligence in Radiotherapy of Nasopharyngeal Carcinoma with Magnetic Resonance Imaging" was retracted in 2023. Reasons: signs of a paper mill; compromised peer review; unreliable results or conclusions.

The specially designed network structure and adaptive convolution can capture different organ features depending on the image resolution in the vertical direction. In the horizontal direction, the feature information captured by the previous layer of the network can be integrated. This hierarchical processing mechanism allows the information to be processed more efficiently in the network.

In medical image segmentation, positive samples only account for a part of the total samples. In loss design, it is necessary to reduce the weight of negative samples in loss in order to alleviate the problem of sample imbalance. We use the focal loss as the loss function of the network, which can balance the performance degradation caused by the difference between positive and negative samples. Formula (2) explains how to calculate the loss value. *p*_*t*_ represents the probability of class T. The number of samples in class *T* and *α*_*t*_, *α*_*t*_ are compression factors to reduce the loss of easily classified samples. *γ* The general value of is set to 5.

(2) $$\begin{array}{c} L\left(p_{t}\right)=-\alpha_{t}{\left(1-p_{t}\right)}^{\gamma }\log\left(p_{t}\right), \end{array}$$

## 5. Experimental Setup and Working Mechanism

Because nasopharyngeal carcinoma endangers many organs and has great differences in shape and volume, we selected 12 main organs (including brain stem, spinal cord, left parotid gland, right parotid gland, left eye, right eye, left temporal lobe, right temporal lobe, throat, left mandibular gland, right mandibular gland, and thyroid) to evaluate the segmentation of the algorithm. In addition, for several small organs (including left optic nerve, right optic nerve, and optic chiasm), AUnet was compared with traditional UNET and DDNN.

The AUnet partitioning model converged on 12 major organs and 3 minor organs simultaneously. The test environment used an Nvidia 2080ti GPU; the entire training process took about 45 hours.

### 5.1. Quantitative Evaluation

In the testing phase, we test all 3D CT images one by one. The input was 3D CT images and the final output was classified at pixel level after which the most likely classification label was the output contour. The results were quantitatively analyzed using similarity coefficient (DSC) and Hausdorff distance (HD) and compared with manual segmentation by physicians. The DSC similarity coefficient was calculated as shown in

(3) $$\begin{array}{c} DS\;C\left(A,B\right)=\frac{2|A\cap B|}{\left|A|+|B\right|}, \end{array}$$

where *A*∩*B* denotes the intersection of A and B.

The article "Application of Artificial Intelligence in Radiotherapy of Nasopharyngeal Carcinoma with Magnetic Resonance Imaging" was retracted in 2023. Reasons: signs of a paper mill; compromised peer review; unreliable results or conclusions.

The HD is calculated as shown in

(4) $$\begin{array}{c} H\left(A,B\right)=\max\left(h\left(A,B\right),h\left(B,A\right)\right), \end{array}$$

where *H*(a, b) denotes the maximum distance between the point in the set A and the set B, denoted as

(5) $$\begin{array}{c} h\left(A,B\right)=\max_{a\in A,b\in B}\left(\min||a-b||\right), \end{array}$$

### 5.2. Results and Observations

The OARs all had DSC values greater than 0.73, with a mean value of 0.86 and HD values within 4.7 mm, with a mean value of 4.0 mm. Among them, eye segmentation had the highest accuracy, with a DSC of 0.93, while spinal DSC values were lower, with a HD of 3.5 mm. The mean values of DSC and HD for AUnet, DDNN, and Unet were over 12 organs (Figures 5 and 6).

The segmentation results of a randomly selected batch of experiments (Figure 7) are presented, thus revealing the performance of the proposed network in this paper. The average segmentation time for automatic segmentation of OARs in CT images of 20 test set patients using the AUnet study model is about 13 seconds, which is a great improvement in efficiency over manual outlining.

The results of this study also showed that the difference between the location of the automatic outline results and the manual outline organs was small (Figure 7). One of the fold cross-validation results is shown in Figure 8. The results showed that the loss function gradually stabilized after about 250 epochs. There was no statistical difference between the automatic segmentation results of AUnet and the manual segmentation results of physicians (*p* > 0.05).

As one of the most popular algorithms for deep learning, deep convolutional neural networks consist of multiple convolutional and pooling layers that can extract multilevel visual features for automatic prediction. These pooling layers will downsample from *x*, *y*, and *z* directions simultaneously, and the head and neck radiotherapy endangered organs contain many small organs, among which such small organs as optic nerve and optic cross take up fewer layers, usually only two to three layers. And after multiple pooling, the features of small organs are easily lost, which makes the segmentation accuracy of small organs not high. This model has a large memory requirement, so a too deep feature extraction network is not used, which may be the main reason for the unsatisfactory segmentation of small organs. In the next study, we will try to design deeper feature extraction structures for comparative analysis to further improve the segmentation performance. Zijdenbos et al. proposed that DSC > 0.7 would indicate high repetition of both and better segmentation.

The article "Application of Artificial Intelligence in Radiotherapy of Nasopharyngeal Carcinoma with Magnetic Resonance Imaging" was retracted in 2023. Reasons: signs of a paper mill; compromised peer review; unreliable results or conclusions.

The quantitative evaluation index (DSC and HD) values of the automatic segmentation accuracy of the test set of small organs and the DSC values of AUnet segmentation were above 0.50 (mean value of 0.61) and the HD values were within 4.0 mm (mean value of 3.4 mm), while the DSC values of small organs were low, but the HD values were only 3.4 mm, which also indicated a high segmentation accuracy. The low DSC values were due to the smaller size of the organ, which led to the lower DSC calculation. Because of the smaller volume of the organ, the AUnet segmentation results of the left optic nerve, right optic nerve, and optic cross have statistical differences from the manual segmentation; however, compared with the traditional Unet and DDNN, there has been a large improvement.

Comparison of the images of the two outlining methods: automatic outlining and manual outlining endangered organ contours basically (Figures 9(a)–9(f)), but with slight gaps, such as large gaps in several layers of the temporal lobe (Figure 9(a)), gaps in the demarcation of the brainstem and spinal cord (Figure 9(b)), and gaps in the outline of the mandible at the level of larger gradients (Figure 9(d)), which could basically achieve the manual outlining effect after minor modifications. The eye, crystal, thyroid, and parotid gland basically meet the requirements.

In addition, the automatic outline time for organ endangerment was statistically close to 60 s/patient, while the manual outline time ranged from 2 to 3 h. Automatic sketching greatly improves the efficiency.

In summary, the application of AccuContour, an artificial intelligence-based automatic outlining software, in the outlining of organs at risk in radiotherapy for nasopharyngeal carcinoma is basically feasible, and the accuracy of the outlining of organs at risk for small volumes is inferior to that of larger volumes, and it can be used in clinical practice with minimal modification by physicians, which can improve the efficiency. It should be noted that the sample size of this study is limited and the results may be biased, and the next step will be to include a multicase study.

The article "Application of Artificial Intelligence in Radiotherapy of Nasopharyngeal Carcinoma with Magnetic Resonance Imaging" was retracted in 2023. Reasons: signs of a paper mill; compromised peer review; unreliable results or conclusions.

## 6. Conclusions

In the treatment of nasopharyngeal carcinoma, with the development and widespread use of intensity-modulated radiotherapy technology, the requirements for the accuracy of imaging technology have become higher and higher. Imaging examinations, such as CT, MRI, and PET, have important applications in the diagnosis, target area determination, efficacy evaluation, and regular follow-up of patients with nasopharyngeal cancer, among which MRI has become the most widely used clinical examination method due to its sensitivity, accuracy, and noninvasiveness. However, due to the insensitivity of conventional MRI to early bone destruction, the artifacts caused by volumetric effect and uneven magnetic field enhancement, which often cause uneven or abnormal signal of skull base bone in conventional MRI, and the long time required for recovery of skull base bone breakage after radiotherapy, conventional MRI has certain limitations in determining skull base bone destruction of nasopharyngeal carcinoma and evaluating its efficacy. Therefore, in the absence of evidence of direct invasion of skull base bone by nasopharyngeal carcinoma lesions, whether the abnormal signal of skull base is tumor invasion, tumor recurrence, and residual tumor and whether it is changed after radiotherapy has become a difficult problem for radiologists and imaging physicians.

In some patients with nasopharyngeal carcinoma, factors such as mild bone cortical invasion in early stages and difficulty in differentiating from reactive bone hyperplasia lead to the difficulty of accurate diagnosis of lesion invasion structure and extent by conventional MRI, and also conventional MRI cannot provide objective quantitative information of invasion, which makes it difficult to accurately outline the target area for clinical radiotherapy. In contrast, DWI sequences are highly sensitive, and when the lesion is confined to the bone marrow without cortical destruction, DWI is more sensitive than nuclide bone imaging. Therefore, the combination of conventional MRI and measured ADC values in this study is beneficial to accurately determine the nature and extent of the lesion. Normal bone tissue includes bone cortex and bone cancellous, and the main component within the bone cancellous is bone marrow. The normal bone marrow consists of red and yellow marrow, and the bone marrow is composed of hematopoietic cells, adipose tissue, water, proteins, and bone trabeculae. The apparent diffusion coefficient ADC, obtained by DWI, reflects the restricted activity of water molecules in bone structures, and its ADC value is significantly lower than that of soft tissue structures. When the nasopharyngeal carcinoma tumor lesion invades the slope, it destroys and alters the normal osteoblasts and bone marrow components, causing bone loss and replacing them with a large number of tumor cells. The difference in ADC values between the invaded slope and normal slope tissue was analyzed to be statistically significant.

The article "Application of Artificial Intelligence in Radiotherapy of Nasopharyngeal Carcinoma with Magnetic Resonance Imaging" was retracted in 2023. Reasons: signs of a paper mill; compromised peer review; unreliable results or conclusions.

The number of cases selected for this study was relatively small, the study time was short, and there were many factors affecting the ADC value measurement results, such as advanced equipment, equipment stability, scanning parameters, scanning time, and physician awareness differences, which made this study somewhat limited. The study has some limitations, and a more in-depth study with a larger sample size is needed to better apply DWI functional imaging technology in clinical practice.

In conclusion, this study concluded that DWI as a functional imaging technique will have a broader application in the diagnosis and treatment of skull base invasion of nasopharyngeal carcinoma.

For preprocessing CT images using adaptive histogram equalization, in this paper, we use end-to-end training to improve modeling efficiency and implement a 3D Unet-based improved network (AUnet), which introduces organ size as prior knowledge into the convolutional kernel size design to enable the network to adaptively extract features of organs of different sizes, thus improving the performance of the model. The DSC (Dice Similarity Coefficient) coefficients and Hausdorff (HD) distances of automatic and manual segmentation are compared to verify the effectiveness of the AUnet network. The average DSC and HD of the test set were 0.86 ± 0.02 and 4.0 ± 2.0 mm, respectively [12].

## Figures and Tables

**Figure 1:** General flow chart of the proposed model.

**Figure 2:** AUnet structure of the proposed model.

**Figure 3:** AUnet details.

**Figure 4:** Schematic diagram of AUnet jump connection.

**Figure 5:** Box plots of DSC similarity coefficients for 12 organs.

**Figure 6:** Box plots of HD values for 12 organs.

**Figure 7:** Nuclear magnetic images.

**Figure 8:** Training loss curve of AUnet.

**Figure 9:** Comparison of automatic and manual outlining of organ endangerment.

## Data Availability

The datasets used and analyzed during the current study are available from the corresponding author upon reasonable request.
